# Research on the Construction of University Public Health Emergency Management System Based on Psychological Counseling Intervention

**DOI:** 10.1155/2022/2033018

**Published:** 2022-01-12

**Authors:** Lingling Zhang

**Affiliations:** Yangzhou Polytechnic Institute, Yangzhou, Jiangsu 225127, China

## Abstract

After entering the information society, all kinds of risks, crises, and conflicts in society are more severe, more sudden, and uncertain than those in agricultural society and industrial society. Under the unexpected events in colleges and universities, college students' psychological crisis, which cannot be dealt with and overcome by conventional methods, arises from their own experiences, psychological endurance, and weak self-awareness. In the face of emergencies, as a talent training base, how to collect information quickly and accurately and make prevention and control plans is directly related to the success or failure of event handling. This study attempts to analyze the characteristics and causes of students' psychological changes in public health emergencies in colleges and universities and puts forward relevant countermeasures, so as to improve the management system of public health emergencies in colleges and universities, improve the ability to effectively deal with and properly handle public health emergencies, and promote the harmonious development of society. In the face of public health emergencies, colleges and universities should enhance the awareness of emergency management of public health emergencies, change the concept of emergency, build an efficient emergency management system, improve the ability and level of emergency management, and ensure the harmony and stability of the school.

## 1. Introduction

With the negative impact of social and industrial development, the frequency of public health emergencies is constantly increasing, and the types of public health emergencies are constantly changing. While enjoying the convenience brought by modern civilization, human beings are constantly facing the challenges of various health hazards [1]. Public emergencies are natural disasters, accident disasters, public health events, and social security events that occur suddenly, cause or may cause serious social harm, and need to take emergency measures to deal with them [2]. With the development of the times, colleges and universities pay more attention to the stability of the school, and the emergency treatment of campus emergencies has been listed as an important work by many colleges and universities [3]. Since the 30 years of reform and opening up, China's economic and social development has made remarkable achievements, but there are also many deep-seated contradictions. People's livelihood problems gradually emerge and accumulate, which became a hidden danger affecting social harmony and stability [4]. In the face of emergencies, as a talent training base for colleges and universities, how to quickly and accurately collect information, develop prevention, and control programs is directly related to the success or failure of event handling [5].

Under the emergencies in colleges and universities, due to their own experience, psychological endurance, weak self-awareness, and other reasons, college students cannot deal with and overcome the psychological crisis by using conventional methods [6]. Once the students have psychological crisis, they will show it in cognition, emotion, behavior, and so on. In order to improve the overall emergency management ability and level of colleges and universities, under the new situation, colleges and universities are required to establish and improve the emergency management system, improve the collaborative operation mechanism of emergency management, strengthen the construction of emergency management team, enhance the ability of emergency material supply, and improve the emergency management level and ability of public health emergencies [7]. This study attempts to analyze the characteristics and causes of students' psychological changes in public health emergencies in colleges and universities and put forward relevant countermeasures, so as to improve the management system of public health emergencies in colleges and universities, improve the ability to effectively respond to and properly handle public health emergencies, and promote the harmonious development of society.

## 2. Definition and Characteristics of Public Health Emergencies in Colleges and Universities

We should improve our understanding of the importance of school mental health education. Students are not only the cognitive body of learning knowledge but also the living body of flesh and blood. Strengthen mental health education and cultivate students' positive, optimistic, upward, and antifrustration psychological quality. Promoting the development of students' sound personality is an inevitable requirement for the implementation of quality education. Schools should cultivate talents with China's education priority development strategy, and the cultivation of talents should start from schools. Sudden public events refer to emergencies that occur suddenly, are unpredictable, may cause loss of personnel and property, bring psychological panic to the parties and have serious harm to social public safety, and need to make decisions in a short time and with incomplete information. Psychological crisis intervention is not a medical behavior, but a programmed psychological first aid. The relationship between psychological crisis intervention and psychotherapy is the same as that of medical first aid to surgery. Giving full play to the advantages of the socialist system with Chinese characteristics in great practice and strengthening and innovating social governance are important channels to enhance China's national governance system and governance capacity [8]. Public health emergencies are group acute events caused by physical, chemical, biological, and other factors, which are sudden, concealed, group, and fearful, and will cause great influence and harm to society. Emergency management of public health emergencies is an important part of practicing the concept of education management and service in colleges and universities, and it is also an important indicator to measure and reflect the overall management ability and level of colleges and universities. Regardless of the nature and scale of the school, the occurrence of unexpected events in colleges and universities will destroy the normal order of school teaching and students' life to varying degrees, affect the reputation of the school in society, and cause extreme panic and confusion in the thoughts and psychology of teachers and students.

Public health emergencies have a direct or indirect impact on people's psychology, showing different characteristics according to people's psychological endurance. At present, although there are different opinions on the concept and connotation of psychological endurance, there are still controversies. More and more scientific research studies show that people's health or diseases can be induced by their social behavior and psychology, and a positive attitude can effectively improve their physiological and psychological immunity, which has an irreplaceable role in modern biomedicine. As an important department of college students' education management and ideological and political education system, when public health emergencies occur, the related safety protection and ideological and political education work carried out by college students' engineering departments is an important support for the prevention and control of public health emergencies in colleges and universities and reflects the coping level of public health emergencies in colleges and universities. In a society with increasingly developed science and technology, people have realized the characteristics of many infectious diseases and prevented and controlled their emergence and spread by scientific means. After the occurrence of the public crisis, the processing time is very urgent. If the judgment is not accurate and the handling is decisive, the consequences will be irreparable, and even the whole school-wide teaching order will be paralyzed, and the impact will be very bad.

According to the scale of the loss caused by the epidemic to the total economic output and then divided by the total labor productivity, the employment loss caused by the epidemic can be calculated. The basic idea can be expressed as follows:

(1) $$\begin{array}{c} L=\frac{\text{GDP}}{\text{GDP}/L}. \end{array}$$

Among them, *L* represents the number of jobs, and GDP represents the gross domestic product. GDP/L is the gross domestic product per labor, that is, the labor productivity of all employees. Expressed by P, the formula (1) can be expressed as

(2) $$\begin{array}{c} L=\frac{\text{GDP}}{P}. \end{array}$$

Using *t*_0_ and *t*_1_ to represent the two periods before and after the epidemic, the change in the number of employment before and after the epidemic ΔL can be expressed as

(3) $$\begin{array}{c} \Delta L=L_{t_{1}}-L_{t_{0}}\\ =\frac{{\text{GDP}}_{t_{1}}}{P_{t_{1}}}-\frac{{\text{GDP}}_{t_{0}}}{P_{t_{1}}P_{t_{0}}}. \end{array}$$

If we simply examine the impact of the epidemic on the number of employment, we need to assume that other factors affecting the economy and employment remain unchanged, and the above formula is simplified to

(4) $$\begin{array}{c} \Delta L=\frac{\Delta \text{GDP}}{P_{t_{0}}}. \end{array}$$

With the improvement of medical and health level, people have become somewhat unfamiliar and forgotten about epidemic infectious diseases and their harms. Sudden emergence of various epidemic diseases often leads to panic and lack of sobriety and calmness. Public health emergencies are accompanied by an increase in the number of patients, especially the death toll. Human beings know little about them, and the epidemic spreads rapidly. It is inevitable that some people will feel uneasy or even panic in a short time. However, some people's MoMo psychology of alienating people in epidemic areas and rejecting those who have recovered from illness, their fear of death in despair and pessimism, and their gloating psychology of seeing others get sick are all abnormal. These psychology and behaviors are not conducive to the prevention and treatment of sudden public health incidents, but will cause greater harm to innocent people, even engender social hostility and trigger social unrest.

## 3. Construction of the Management System of Public Health Emergency in Colleges and Universities

### 3.1. Strengthening the Consciousness of Emergency Management in Colleges and Universities

In public health emergencies, paying attention to the health status of college students and ensuring their personal safety are the top priority of all the works of the relevant student departments in colleges and universities. After the crisis, students hope that their lives can be restored to normal as soon as possible, and they are eager for the understanding and support of others, which provides a basis for crisis intervention. The occurrence of crisis events is unpredictable, so it is particularly important for colleges and universities to establish a perfect psychological crisis intervention mechanism in order to effectively deal with crisis events [9]. Counselors should talk with students in a targeted way, help students solve psychological confusion in time, and find abnormal students who should immediately give feedback to the school mental health consultation center. In the face of public health emergencies, people with good social and psychological qualities, whose extraordinary understanding and calm are invisible resources, can inspire people to unite and overcome disasters.

Emergency management should do a good job of prevention from the source of emergencies, nip in the bud, and improve the handling mechanism and guarantee mechanism. College administrators should have a sense of urgency, make emergency plans well, and strengthen the exercise of emergency events, so that they can calmly deal with unexpected problems and avoid chaos in times of crisis. The interactive relationship of students' social development is shown in Figure 1.

In order to enhance the important understanding of college administrators on emergency management of public emergencies and fundamentally solve the problem of neglecting ideological understanding, it is necessary to regularly educate and train college administrators on emergency management, improve the level of theoretical knowledge, and strengthen the forward-looking handling of emergency management of public emergencies. In the sensitive period of public health emergencies, the communication between governments at all levels, departments, government departments, and medical departments must be smooth, high speed and convenient, so as to make government decrees unimpeded. The government must provide open and transparent information, manage information scientifically and effectively, and enhance the reliability, speed, and validity of news dissemination. After an incident occurs, the emergency plan should be started quickly, the specific situation of the superior department should be reported, the situation should be controlled to the best of its ability, the grade, severity, change trend, and influence range of the accident should be evaluated quickly, and the information should be reported in time to avoid unnecessary panic.

### 3.2. Improving the Emergency Management System in Colleges and Universities

Public emergencies will have different impacts on different individuals, which require different group counseling for different problem groups. When an emergency happens, it is also very important to manage emergency materials, so it is important to reserve emergency materials in peacetime. Colleges and universities should combine their own situation, actively improve the emergency call, integrate existing manpower and financial resources, and record the corresponding emergency materials. The financial department is responsible for the reserve funds, while the campus construction department is responsible for putting the reserves in place [10]. Good social psychological endurance needs long-term education and training. At present, our school education generally lacks life education courses and basic knowledge and skills education on disaster prevention and avoidance. Therefore, it is suggested that local education authorities should set up life safety courses compulsorily, continuously, and moderately according to local regional characteristics. In the face of public health emergencies, human beings should learn to tide over difficulties hand in hand. Any deliberate avoidance, escape, or concealment is immoral.

Although the outbreak of college students' psychological crisis has the characteristics of suddenness and urgency.  Figure 2 shows the evolution structure of college students' psychological crisis.

In order to deepen the safety awareness of all teachers and students, ensure that all teachers and students can escape quickly, safely, and orderly in the face of some emergencies, and to minimize the losses caused by emergencies, colleges and universities should regularly organize teachers and students to carry out safety emergency evacuation drills on fire prevention and earthquake prevention. Exercises close to the real situation can restore emergencies to a great extent. It is necessary to use modern information network technology to establish a data monitoring system for emergency management, focus on building an information monitoring system involving all employees, combine traditional and modern methods, establish an information sharing mechanism, upload students' health information in time, analyze and screen the information of sick students, and provide accurate basis for prevention and treatment. Colleges and universities need to issue normative documents, refine detailed rules, strengthen emergency knowledge education for teachers and students, and help teachers and students improve their ability to cope with crises, such as offering emergency management courses, holding regular emergency management knowledge training lectures, and holding regular emergency drills.

## 4. Conclusions

Regardless of the nature and scale of the school, the occurrence of emergencies in colleges and universities will destroy the normal teaching order and students' life in varying degrees, affect the reputation of the school in the society, and cause extreme panic and confusion in the thoughts and psychology of teachers and students. Counselors should have targeted conversations with students, timely help students solve their psychological confusion, and students who find abnormalities should immediately give feedback to the school mental health counseling center. Colleges and universities should use modern information network technology to establish an emergency management data monitoring system, focus on building an information monitoring system with the participation of all staff, upload students' health information in time, and analyze and screen the information of sick students, so as to provide accurate basis for prevention and treatment. In the face of public health emergencies, colleges and universities should enhance the awareness of emergency management of public health emergencies, change the concept of emergency, build an efficient emergency management system, improve the ability and level of emergency management, and ensure the harmony and stability of the school.

## Figures and Tables

**Figure 1:** Interactive relationship between students' social development.

**Figure 2:** The evolutionary structure of college students' psychological crisis.

## Data Availability

The data used to support the findings of this study are included within the article.
